# Controlled Hypotension Combined with Femoral Nerve Block for Knee Replacement without Tourniquet

**DOI:** 10.1155/2021/3219337

**Published:** 2021-12-09

**Authors:** Liangming Wang, Yiqiang Zheng, Xiaolu Zhang, Qingfeng Ke

**Affiliations:** Department of Joint and Trauma Surgery, The Second Affiliated Hospital of Fujian Medical University, Quanzhou, China

## Abstract

In the process of knee replacement surgery, the use of tourniquet technology for hemostasis is the most common method. But the adverse reactions of tourniquets in knee replacement surgery have become more prominent in recent years. More and more scholars have begun to advocate the optimization of the use of tourniquet technology, thereby controlling the use of tourniquet technology. In this study, 125 patient cases were randomly divided into four experimental groups for comparative analysis. The two sets of variables are whether to use tourniquet during surgery and use intravenous analgesia or nerve block analgesia. Studies have shown that when using a tourniquet for knee replacement surgery, the chance of hidden blood loss increases after use. The tourniquet was not used during the operation, the patient's thighs were swollen, and postoperative pain was reduced. Compared with intravenous analgesia, knee joint replacement with uncontrolled tourniquet combined with femoral nerve block has a better analgesic effect and can effectively relieve pain after knee replacement. Therefore, under the method of controlled hypotension combined with femoral nerve block, TKA surgery without using tourniquet technology is more conducive to early health recovery and pain relief after TKA surgery, as well as functional exercise and knee joint recovery during postoperative recovery.

## 1. Introduction

TKA has widely been used in medical clinical treatment in recent decades. TKA surgery isveryeffective for the advanced management of knee arthritis, and it is arelativelymature and complete surgical method[1]. With the maturity of surgical operation technology and the development of the prosthetic material industry in recent years, patients with knee arthritis will generally choose knee replacement surgery to cure inflammation in the late stage of arthritis[2]. The tourniquet is a common method of hemostasis in clinical research,andit isveryeffective in reducing bleeding during surgery. The tourniquet not only reduces the amount of bleeding during surgery, but also has a good effect in providing a clean and clear surgical field of view;however, in recent years, with the theoretical point of view on the restrictive use of tourniquets[3], more and more scholars have begun to call for optimization and upgrading of tourniquet use methods.

Reducing the amount of bleeding is an important indicator during the operation of TKA. At this time, the use of tourniquet can not only reduce the amount of bleeding, but also provide a clear vision and reduce the bleeding of the bone surface. The use of tourniquets during surgery allows the bone cement component of knee surgery to penetrate better into loose bones and thus can fit the bone surface more firmly [4]. In addition, the tourniquet can reduce the amount of bleeding during the operation, thereby providing the operator with a clear surgical field of vision, cleaner bone cement, and a better bone interface. Therefore, it is widely used in clinical applications of TKA. However, it is currently controversial whether the use of tourniquets can really reduce the total blood loss during the perioperative period of TKA and improve the effect of recovering from the healing period after surgery [5]. The use of tourniquets during surgery may increase the chance of postoperative complications [6]. The application of the tourniquet technique in the TKA process will reduce the pain and swelling of patients during postoperative recovery, speed up postoperative recovery time, and affect the changes in total operation time and total blood loss. In recent years, these claims have been increasing in TKA surgery research. Is the length of tourniquet used related to the occurrence of various complications after surgery [7]? The application methods of tourniquets in replacement surgery have been roughly divided into three categories in recent years. Compared with the frequency of using tourniquets during surgery, they are divided into three situations: the tourniquet is used throughout the procedure, some tourniquets are used, and no tourniquets are used. There are great disputes among experts and scholars on the three types of application methods [8]. Experts and scholars who adhere to the concept of rapid rehabilitation believe that if the use of tourniquets is reduced or not used during TKA surgery [9], it may reduce ischemia-reperfusion injury and thrombosis during surgery [10]. This study proposes a new method of use: combining controlled hypotension with femoral nerve block and using tourniquet only when using bone cement [11].

Although the tourniquet brings some convenience, it also causes some postoperative complications, such as site damage caused by ischemia-reperfusion, local swelling, paralysis, and pain in the tourniquet work area [12]. Therefore, TKA surgery also has disadvantages such as greater trauma and more perioperative blood loss. How to apply tourniquet in the surgical process to maximize the benefits of the tourniquet application during surgery has become a hot research in recent years. Therefore, this study proposes a new method of use: the application of tourniquet under controlled hypotension combined with femoral nerve block [13]. By comparing the impact of the rehabilitation efficiency of different hemostatic methods, the best solution for using a tourniquet in knee replacement surgery is sought. The research team believes that if the reduction or restriction of the use of tourniquets during TKA surgery may reduce the damage caused by the use of tourniquets during and after surgery. The use of a balloon tourniquet during surgery is a routine operation for joint surgeons at home and abroad [14]. It can provide a clear surgical field of view, shorten the operation time, reduce the amount of bleeding during the operation, and provide a good bone cement interface. However, at the same time, the use of tourniquets during surgery can cause discomfort and may even cause pain, venous thrombosis, and muscle and nerve damage [15]. Whether the tourniquet is used during TKA surgery has many different opinions in the medical community [16]. This article uses a systematic review method to analyze the randomized control parameters of tourniquet used in TKA surgery to explore the effect of controlled blood pressure combined with femoral nerve block tourniquet on TKA clinical practice [17].

## 2. Research Methods

### 2.1. Patients' Information

After the approval of the relevant departments of the hospital and the consent of the patient and his family, the research project includes patients with unilateral TKA unilateral limbs who were seen in the hospital from March 2018 to January 2020, regardless of gender, age from 50–80 years, ASA I–III, and NYHA I–III. Some cases that could not be studied were screened, and some cases that had serious complications after TKA surgery or could not be completed due to other reasons and could not complete the data standards required for this surgical study were screened and excluded. We exclude patients with a history of allergy to related surgical drugs, mental illness, cognitive dysfunction, or cardiovascular and cerebrovascular diseases, and other factors that affect the patient's medical experience and safety. Using random allocation, the software automatically divides the selected patients into four groups: the first group's surgical method is TKA surgery using tourniquet combined with vein-controlled analgesia; the second group used tourniquet technique before TKA operation and analgesia with femoral nerve block after operation; the third group used TKA operation without using tourniquet technology and cooperates with intravenous analgesia to reduce postoperative pain; and the fourth group's surgical method is TKA surgery without using tourniquet technology combined with femoral nerve block technology to relieve pain after surgery [18].

### 2.2. Tools

All patients followed the routine fasting and fasting requirements before surgery and routinely monitored HR, SpO_2_, invasive arterial pressure, and depth of EEG consciousness after entering the operating room. In the first and second experimental types, patients with TKA surgery use tourniquet technique on the affected limb, and the pressure of the tourniquet will increase the contraction pressure of the affected limb by 100 mmHg. In the second and fourth groups of surgical experiments, the femoral nerve block was used for anesthesia induction during TKA surgery, and the third and fourth patients underwent TKA surgery without using tourniquet technique. Anesthesia induction was performed in the third and fourth groups of surgery: propofol 1.5 mg/kg, sufentanil 0.5 *μ*g/kg, midazolam 0.5 mg/kg, and rocuronium 0.8 mg/kg. After the induction is completed, the following doses should be maintained during the operation: propofol 3 mg·kg^−1^·h^−1^, remifentanil 0.2 *μ*g·kg^−1^·min^−1^ continuous intravenous pump input, and continuing to inhale 1% sevoflurane and rocuronium 15 mg to maintain muscle relaxation by intermittent intravenous bolus injection. About thirty minutes right before the operation, the muscle relaxant injection was stopped. At the same time, in order to suppress postoperative vomiting, parecoxabine 50 mg analgesia and tropisetron 3 mg were administered, and the suture operation was started after the use of sedative drugs was stopped. After the operation of the first group of patients, continuous intravenous self-controlled analgesia was performed in order to alleviate the suffering of the patients. This method is referred to as patient controlled intravenous analgesia (PCIA). Its formula is tramadol 10 mg/ml, flurbiprofen axetil 1.25 mg/ml, total volume 80m, background dose 1 ml/h, single injection dose 1.5 ml; lock-in time: 15 min. The second group performed the operation of self-controlled analgesia of the femoral nerve block after operation. This method is referred to as patient controlled nerve block analgesia (PCNA). Its formula is concentration of ropivacaine is 0.125%, the total volume is 300 ml, flurbiprofen axetil is 1.25 mg/ml, total volume is 80m, background dose is 5 ml/h, and single injection dose is 5 ml; lock-in time: 45 min. The PCIA method was used for analgesia in the third group after the operation, and the content of the PCIA formula was the same as that of the first group. The PCNA method was used for analgesia in the fourth group after the operation, and the content of the PCNA formula was the same as that of the second group. The time and blood loss of the patients in the TKA operation were used as observation indicators for statistical analysis The total blood loss data Hb(g/L) on the day before the operation and the day after the operation are calculated as follows:

(1) $$\begin{array}{c} \text{total blood loss}=\left(\text{Hb before surgery}-\text{Hb after surgery}\right)\times \text{body weight}\left(\text{kg}\right)\times 7.5. \end{array}$$

The circumference of the upper third of the patient's thigh was measured on the day before the start of the TKA operation and one, two, and three days after the end of the operation. Peripheral venous blood of the affected limb was collected to determine the WBC count, NEUT%, and CRP concentration data. The patient's affected knee joint activity (AROM) was evaluated one day before the operation, and one, two, three, and seven days, and three months after the operation. One day before surgery, and one, two, three, and seven days, and three months after surgery, using the VAS, pain during rest and activities was measured [19], and the scoring standard was set as follows: 0 points, painless; and 10 points, unbearable pain [20]. This study used the MoCA scale to evaluate cognitive function [21], and continuous data monitoring and statistical analysis were performed on the day before the operation, the first day after the operation, the second day after the operation, and the third day after the operation. In the MoCA scale, a total of eight data display performances such as visual space, executive function, naming, and memory can be listed.

### 2.3. Analysis Method

Using the statistical analysis method of this study [22], the collected data information is analyzed and processed statistically by using SPSS 19.0 statistical software. If the measurement data after analyzing the data conform to the normal distribution law, then the data are expressed in the form of mean and standard deviation (*x* ± *s*). Two-way ANOVA was used as the standard to compare the analysis methods between the two groups of data. The SNK-q test standard was used as the method standard for the comparison between the two sets of data [23]. We use the SNK-q test standard as the method standard for pairwise comparison between the two sets of data. We use the LSD-t method to test the data and compare the values at different time points in the data set. The LSD-t method was used to test the data, and the numerical values at different time points in the dataset were compared. The counting data were tested by *χ*^2^. When *P* < 0.05, it was indicated that the statistical standard was met, and the data standard had statistical significance.

## 3. Results

Among the clinical cases of surgery that covered 128 patients with knee arthritis, only 125 were effective cases in this study. A total of 3 patients in the 128-patient case suffered from other serious complications after surgery and were transferred to the respiratory medicine department and excluded from the screening criteria. A total of 125 TKA patients participated in the completion of this study, and there was no statistical difference between patients' characteristics, such as age, gender, occupation, and education level. Within the period of postoperative recovery in the hospital where the operation was performed, there was no statistical difference between the four groups of patients. The difference in the time spent during the TKA operation was not much different in the data analysis of the groups of patients studied, so it was not statistically significant. During the TKA operation, the bleeding volume in the first and second groups was significantly lower than that in the third and fourth groups (*P* < 0.05). However, the total blood loss of the first and second groups was higher than that of the third and fourth groups (*P* < 0.05), as shown in Figure 1.

On the 1st, 2nd, and 3rd days after the operation, the thigh circumference of the first and second groups increased more than that of the third and fourth groups (*P* < 0.05). Since the data difference between the first and second groups is not statistically significant at different points in time, and the data difference between the third and fourth groups is not statistically significant, this difference can be ignored, not counted, and therefore not considered to be the parameters of this study, as shown in Figure 2.

Compared with the day before the TKA operation, the WBC data and NEUT% values of each group of patients on the first day after the operation had a significant increase (*P* < 0.05). At the same time, the data between the groups is not very different, so there is no statistical significance. On the first day, the second day, and the third day after the TKA operation, the CRP concentration in the first and second groups was lower than that in the third and fourth groups (*P* < 0.05). The CRP concentration data between the first group and the second group were not different at different time points, and the CRP concentration data between the third group and the fourth group were not different at different time points, so the data were not statistically significant, as shown in Table 1.

According to the statistical analysis of the data on first and second days after the TKA operation, the AROM of the second and fourth groups is greater than that of the first and third groups (*P* < 0.05). At three and seven days and three months after the operation, there was not much difference between the four groups, so there was no statistical significance. Because at different time points, the difference in AROM values between the first and third groups and between the second and fourth groups is not statistically significant, it is ignored and not considered the object, as shown in Figure 3.

On the first day and second day after surgery, the VAS scores of the first group were higher than those of the second, third, and fourth groups (*P* < 0.05). The VAS scores of patients at rest in the second group, the third group, and the third group were not statistically different, so they were ignored and not considered the study object. The VAS score data of the third group of clinical cases were higher than those of the second and fourth groups (*P* < 0.05). The difference between the first group and the second group is not statistically significant, so it is ignored, and three days and seven days, and three months after the completion of the operation, the VAS scores were not significantly different between the four groups during the rest and activities through different surgical protocols, so there was no statistical significance, as shown in Table 2.

Compared with before surgery, the MoCA scores of the third and fourth groups were significantly lower on the first day after surgery (*P* < 0.05). The MoCA scores of the first and second groups were significantly lower than those of the third and fourth groups, which is obvious (*P* < 0.05). There is no statistical difference between the first and second groups and between the third and fourth groups, so it is ignored. On the second and third days after the operation, there was no statistical difference in the MoCA scores between the four groups of patients, so they were ignored and not considered the subjects of this study. Within three days after surgery, the total incidence of cognitive impairment in the first and second groups was significantly lower than that in the third group, and the difference was even more significant in the fourth group (*P* < 0.05). The data study found that within three days after TKA surgery, the total incidence of PONV in the first and third groups was lower than that in the second and fourth groups (*P* < 0.05), as shown in Figure 4.

## 4. Discussion

In order to reduce the amount of bleeding during the operation during the TKA operation, the tourniquet technique is often used. The use of the tourniquet technique can provide conditions for the hardening of bone cement. Although there will be a small amount of bleeding and the surgery area is slightly blurred, it will not hinder the operation. Therefore, when performing TKA surgery without tourniquet, the clarity of the surgical field of vision does not affect the surgery. In the above study, it was found that the amount of bleeding in the operation after the use of the tourniquet during the TKA operation was significantly reduced, but the total blood loss within one day after the operation of the patient after one day would be greater than that during the operation without the tourniquet of patients. The causes of complications such as ischemia, nerve damage, and swelling of the lower limbs have little to do with the use of tourniquets, and the use of tourniquets during surgery may affect postoperative recovery. The data of this study showed that, under the control of the tourniquet pressure and time, the lower limb limbs will swell for more than three days after guarding. Similarly, when using a tourniquet to stop bleeding, it will cause muscle strain, increase muscle fiber cross section, structural abnormalities and reduced function, and other symptoms for several months. Whether it will affect the recovery after TKA surgery in the future is uncertain. The results of the joint mobility values of the patients who were followed up for three months showed that there was no statistical significance for the use of tourniquet. The surgical method without the tourniquet technique in TKA surgery was performed on the patients for one year after TKA. The data in the tracking search show that there is not much difference between the long-term recovery efficiency of patients who do not use tourniquet technology and those who use tourniquet in TKA surgery. In contrast, the use of tourniquets during surgery is more conducive to the early recovery of surgical patients, and there is no significant difference in long-term effects. After the operation of total knee replacement surgery, because of the growth and recovery of a new tissue after the replacement of the knee joint, the affected patient's limb usually suffers from swelling and severe pain. When the tourniquet is used for surgery, it will aggravate severe pain, which will affect the patient's physical recovery after surgery and affect the exercise and recovery of the knee joint. In order to alleviate the severe pain after the operation in total knee replacement surgery, it is recommended that the tourniquet should not be used or the use of tourniquet should be restricted during the postoperative procedure. And the postoperative analgesia program can choose controlled hypotension combined with femoral nerve block technology for analgesia, so as to alleviate the strong pain and discomfort caused by TKA surgery to the patient. The degree/amplitude of blood pressure reduction should be comprehensively measured with reference to many indicators such as electrocardiogram, heart rate, pulse pressure difference, and central venous pressure. For ordinary patients, reducing the original blood pressure by 30% can reduce bleeding, reduce bleeding, and promote surgery without causing serious complications.

This study points out that the use of controlled blood pressure reduction combined with femoral nerve block without tourniquet technique in TKA surgery is more conducive to pain relief at rest after surgery. Patients using tourniquets had poor analgesic effects in the early stage of surgery, and patients using PCNA had significantly lower VAS scores than PCIA in two days. It shows that the analgesic effect is good and it is beneficial to the recovery of the affected limb after operation. Because after the PCNA analgesia operation, the patient's pain is lighter, so the PCNA analgesia technology is more effective than the PCIA two analgesia methods. Therefore, the analgesic method of using PCNA during TKA surgery is more conducive to the early recovery of patients after TKA surgery. In the course of this study, the WBC and NEUT% values both increased and basically returned to normal after two days. This study shows that the change in the NEUT% value is not related to whether the tourniquet technique is used, and is associated with postoperative limb pain not much related to postoperative recovery. This study shows that, within a few days after the end of TKA surgery, the patient's CRP index continues to increase and is above average. And the data detected within three days after the operation showed that the CRP index is still slightly higher than the average level. Persistent inflammation is one of the causes of postoperative cognitive impairment, and it mostly occurs in the first three days after the operation and the data show that the outbreak rate is higher on the first day after the operation. The high incidence of cognitive function may be related to inflammation, but the specific reasons need to be investigated.

## 5. Conclusion

In summary, when the controlled blood pressure reduction combined with femoral nerve block technique is used without a tourniquet in TKA, the degree of swelling and pain of the thighs after surgery was lower than that of patients using tourniquet technique. The analgesic effect of the tourniquet-free method under continuous femoral nerve block is far more effective than intravenous analgesia and can significantly relieve the pain after knee replacement surgery. Therefore, under the method of controlled blood pressure lowering combined with femoral nerve block, surgery without tourniquet is more conducive to the early rehabilitation of patients and pain relief after TKA surgery. At the same time, it also has a significant effect on the functional exercise during the recovery period and the recovery of the knee joint activity after the operation.

## Figures and Tables

**Figure 1:** Comparison of operation time and bleeding volume of four groups of patients.

**Figure 2:** Thigh swelling in the four groups of patients: comparison of thigh circumference.

**Figure 3:** Comparison of AROM of knee joints in four groups at different time points.

**Figure 4:** Comparison of MoCA scores of four groups of patients at different time points, cognitive impairment, and PONV occurrence within 3 days after surgery.

**Table 1:** Comparison of AROM of knee joints in the four groups at different time points.

Index	Group	Number of cases	The day before surgery	1 day after surgery	2 days after operation	3 days after surgery
WBC (10⁹)	1	28	5.5 ± 1.1	10.5 ± 2.4	6.7 ± 1.9	6.1 ± 1.7
	2	30	6.0 ± 1.3	9.8 ± 2.1	6.1 ± 1.5	6.3 ± 1.4
	3	28	5.3 ± 1.4	13.1 ± 2.9	5.2 ± 1.4	5.1 ± 1.6
	4	39	5.8 ± 2.1	13.2 ± 3.4	5.9 ± 2.3	5.7 ± 2.2

NEUT (%)	1	28	55.9 ± 8.4	86.1 ± 11.1	73.1 ± 18.1	66.6 ± 11.1
	2	30	59.6 ± 9.4	81.9 ± 12.4	73.1 ± 17.2	64.3 ± 10.2
	3	28	59.7 ± 7.5	86.9 ± 11.8	69.9 ± 16.6	62.3 ± 11.4
	4	39	68.2 ± 8.8	88.6 ± 15.4	68.9 ± 17.9	66.1 ± 10.9

CRP (mg/L)	1	28	2.9 ± 0.4	18.2 ± 9.1	58.9 ± 11.9	36.3 ± 5.4
	2	30	5.3 ± 1.6	39.1 ± 10.5	59.2 ± 14.1	42.3 ± 9.1
	3	28	4.5 ± 1.5	49.1 ± 9.4	58.5 ± 13.6	56.3 ± 10.4
	4	39	4.5 ± 0.5	53.1 ± 12.8	89.6 ± 16.4	66.7 ± 11.1

**Table 2:** Comparison of VAS scores of four groups of patients at rest and at different time points.

Status	Group	Number of cases	The day before surgery	1 day after surgery	2 days after surgery	3 days after surgery	7 days after surgery	3 months after surgery
At rest	1	28	1.1 ± 0.2	4.5 ± 1.5	3.8 ± 0.8	2.4 ± 0.1	1.4 ± 0.3	0.7 ± 0.3
	2	30	1.2 ± 0.1	2.3 ± 0.2	22 ± 0.5	2.5 ± 0.1	1.3 ± 0.4	0.5 ± 0.4
	3	28	1.4 ± 0.2	2.5 ± 0.2	2.4 ± 0.5	2.6 ± 0.2	1.4 ± 0.4	0.3 ± 0.2
	4	39	1.5 ± 0.2	2.5 ± 0.5	2.6 ± 0.2	2.3 ± 0.5	1.8 ± 0.2	0.8 ± 0.2

When active	1	28	1.7 ± 0.4	4.3 ± 1.5	4.5 ± 1.2	3.0 ± 0.1	1.3 ± 0.3	0.4 ± 0.2
	2	30	1.8 ± 0.3	3.4 ± 1.4	3.1 ± 1.0	2.9 ± 0.5	1.7 ± 0.5	0.9 ± 0.3
	3	28	2.1 ± 0.4	4.8 ± 1.1	4.2 ± 0.5	2.8 ± 0.8	1.9 ± 0.5	1.0 ± 0.3
	4	39	2.0 ± 0.3	3.1 ± 1.4	2.0 ± 0.8	2.6 ± 0.5	1.2 ± 0.8	0.7 ± 0.1

## Data Availability

The datasets and codes of this article are available from the corresponding author upon request.
